RETRACTED

# The cross-talk between DDR1 and STAT3 promotes the development of hepatocellular carcinoma

**DOI:** 10.18632/aging.103482

**Published:** 2020-07-27

**Authors:** Ye Lin, Haosheng Jin, Xianqiu Wu, Zhixiang Jian, Xiongfeng Zou, Jianfeng Huang, Renguo Guan, Xiangling Wei

**Affiliations:** 1 Department of General Surgery, Guangdong Provincial People's Hospital, Guangdong Academy of Medical Sciences, Guangzhou,Guangdong Province, China; 2 State Key Laboratory of Oncology in Southern China, Collaborative Innovation Center for Cancer Medicine, Department of Experimental Research, Sun Yat-Sen University Cancer Center, Guangzhou, Guangdong Province,China

**Keywords:** hepatocellular carcinoma, DDR1, STAT3, EMT, glutamine metabolism

## Abstract

Objective: To investigate the function of discoidin domain receptor 1 (DDR1) in hepatocellular carcinoma (HCC) and to further clarify the underlying mechanism.

Results: DDR1 was significantly increased in HCC tissues and cells, which was related to clinical staging and prognosis of HCC. Upregulation of DDR1 promoted EMT and glutamine metabolism in HCC cells, while loss of DDR1 showed the opposite effects. STAT3 bound with the promoter of DDR1, and facilitated the phosphorylation of STAT3. In turn, activation of STAT3 increased the expression of DDR1. Silencing of STAT3 removed the promoting effect of DDR1 on proliferation, migration and invasion of HCC cells. The in vivo tumor growth assay showed that the cross-talk between DDR1 and STAT3 promoted HCC tumorigenesis.

Conclusions: Our research revealed the positive feedback of DDR1 and STAT3 promoted EMT and glutamine metabolism in HCC, which provided some experimental basis for clinical treatment or prevention of HCC.

Materials and methods: The mRNA expression of DDR1 was detected by qRT-PCR. CCK8 assay, wound healing assay and transwell assay were used to detect the DDR1/ STAT3 function on proliferation, migration and invasion in HCC cells. Western blot was used to calculate protein level of DDR1, STAT3, epithelial-mesenchymal transition (EMT) related proteins.

## INTRODUCTION

Hepatocellular carcinoma (HCC) is the most common primary liver tumor [1]. The histological origin of HCC is relatively simple, but HCC is characterized by high degree of malignancy, strong invasiveness, multiple foci, easy recurrence, metastasis, and poor prognosis [2]. After the efforts of many scholars, although the effect of HCC treatment has improved, the 5-year recurrence rate is still about 60% [3]. The high mortality rate caused by the high recurrence rate makes HCC the second among all cancer mortality rates in China [4]. It has been recognized that the extremely strong invasion and metastasis ability of HCC is the essential factor affecting the recurrence of patients [5]. However, the specific mechanism of HCC invasion and metastasis is unknown at present. Elucidating the mechanism of HCC invasion and metastasis will help to discover new molecular targets, enrich the diagnosis and treatment of HCC, and improve the prognosis of HCC patients.

RETRACTED

Discoidin domain receptors (DDRs) are members of the receptor tyrosine kinase (RTK), including DDR1 and DDR2 [6]. Current research shows that DDR1 is closely related to malignant behavior of tumors [7], and its main function is to regulate collagen synthesis and degradation, enzyme activity, and monitor the formation of extracellular matrix [8]. The role of DDR1 in the malignant biological behavior of tumors has gradually attracted the attention of the medical community in the past two years. In our previous study, we have found that DDR1 was significantly increased in tumor tissues of patients with early recurrence after HCC (<1 year) compared with those with non-early recurrence (> 2 years) [9], suggesting that DDR1 might be a key factor for early recurrence in patients with liver cancer. Recent research indicates that DDR1 is highly expressed in many tumor cells, suggesting that DDR1 plays an important role in the malignant biological behavior of such tumor cells, especially in the process of tumor invasion and metastasis [10, 11]. Interestingly, EMT (epithelial- mesenchymal transition) plays an important role in tumor migration and invasion [12–14]. However, there are few studies on DDR1 and HCC invasion and metastasis

Studies show that glutamine can be used as a raw material for biosynthesis during cell growth and division [15, 16]. Glutamine provides both carbon and nitrogen sources, both of which can be used for the biosynthesis of amino acids, fatty acids, purines, and pyrimidines to support cancer cell biosynthesis, energy metabolism, and intracellular homeostasis, and promote tumor growth [17]. Under nutrient deficient conditions, cancer cells can also obtain glutamine by breaking down large molecules [18]. Tumors can maintain redox balance through glutamine metabolism and fight against oxygen free radical damage inside and outside cells [19]. More importantly, the study found that under hypoxic conditions, glioma cells participate in tumor cell biosynthesis and energy metabolism by taking up a large amount of glutamine [20]. Therefore, glutamine metabolism is of great significance in maintaining the malignant potential of tumor cells.

In addition to the regulation of various upstream signaling pathways, glutamine metabolism can also participate in regulating the activities of multiple signaling pathways [21, 22]. It is worth noting that STAT3 (signal transducer and activator of transcription 3) is a protein family that exists in the cytoplasm and can be transferred into the nucleus to bind to DNA after activation [23]. It has dual functions of signal transduction and transcriptional regulation [24]. After STAT3 is activated, it enters the nucleus and regulates the expression of various genes [25]. However, no research has reported whether STAT3 can affect the expression of DDR1 gene. Thus, in present study, we focused on the function of DDR1 in HCC, and to further clarify the regulation of the cross-talk between DDR1 and STAT3 on EMT and glutamine metabolism.

RETRACTED

## RESULTS

### The expression of DDR1 in HCC tissues and cells

To clarify the role of DDR1 in HCC progression, we first detected DDR1 expression in HCC tissues and cell lines. We collected adjacent tissues and cancerous tissue from 15 patients diagnosed with HCC. qRT-PCR was performed to test DDR1 level. We found that DDR1 was up-regulated in cancerous tissue than that in adjacent normal tissues (Figure 1A). We then analyzed the expression level of DDR1 in patients with different grades of HCC. Interestingly, the expression level of DDR1 was positively correlated with the tumor grade (Figure 1B). According to the median expression level of DDR1 in Figure 1A, the level of DDR1 in HCC tissues was divided into low expression and high expression. Kaplan-Meier curves were used to compare the total survival of patients with low and high expression of DDR1. The 7-year survival rate of HCC patients with high expression of DDR1 was significantly lower than low expression patients (Figure 1C). Meanwhile, we detected the level of DDR1 in human hepatocyte (HH) and HCC cell lines Hep3B, HepG2, SK-Hep-1 and SNU-182. The results showed that DDR1 was increased in serious of HCC cells (Figure 1D and 1E). It is worth noting that the expression of DDR1 was the highest in SNU-182 and the lowest in Hep3B. The results indicated that DDR1 might play a key role in HCC progression.

**Figure 1:** **Expression of DDR1 in HCC tissue and cells.** (**A**) The expression of DDR1 in clinical HCC tissues (n = 15) and adjacent normal tissues (n = 15) determined by qRT-PCR (**p<0.01). (**B**) Another HCC tissues from patients with tumor grade I (n = 8), grade II (n = 8) and grade III (n = 8) were collected, and the expression of DDR1 in was measured by qRT-PCR (*p<0.05). (**C**) The overall survival of HCC patients with low or high expression of DDR1 in HCC tissues were assessed by Kaplan-Meier survival analysis (n = 15, *p<0.05). qRT-PCR assay (**D**) and western blot (**E**) analyzed the expression of DDR1 in human hepatocyte (HH) and HCC cell lines Hep3B, HepG2, SK-Hep-1 and SNU-182 (n = 6, *p<0.05 vs HH).

RETRACTED

### Upregulation of DDR1 promotes EMT and glutamine metabolism in Hep3B cells

As shown in Figure 1D and 1E, Hep3B cells own the lowest expression of DDR1, and we chose Hep3B to force DDR1 expression. We transfected into DDR1 plasmid or NC into Hep3B cells, and qRT-PCR analysis was performed to determine DDR1 transfection efficiency (Figure 2A and 2B). Then, CCK-8 assay showed that overexpression of DDR1 significantly promoted growth rate at 48h and 72h than cells transfected with NC in Hep3B cells, respectively (Figure 2C). Migration and invasion are the key processes for cancer progression, we then tested the role of DDR1 on migration and invasion ability in Hep3B cells. The wound healing suggested that DDR1 increased the wound healing area, which exhibited a higher migratory ability in DDR1 transfected cells (Figure 2D). Transwell assay was used to test invasive ability. The results showed that DDR1 significantly facilitated the cell invasive ability (Figure 2E).

**Figure 2:** **DDR1 promotes EMT and glutamine metabolism in Hep3B cells. DDR1 plasmid or NC was transfected into Hep3B cells.** The expression of DDR1 was determined by qRT-PCR (**A**) and western bolt (**B**) (n = 6, *p<0.05). (**C**) CKK-8 assay was used to examine the cell growth at 0, 24, 48 and 72 h (n = 10,*p<0.05). (**D**) Wound healing assay was used to detect cell migration (n = 6, *p<0.05). (**E**) Transwell assay was performed to check cell invasive ability (n = 6, *p<0.05). qRT-PCR (**F**) and western blot (**G**) were used to test the expression of EMT related genes: Vimentin, N-cadherin and E-cadherin (n = 6, *p<0.05). The protein expression of glutamine metabolism related genes: GLUD1, GLS1 and SLC1A was determined by western blot (**H**) and immunofluorescence (**I**) (n = 6, *p<0.05).

Numerous evidences revealed the vital role of EMT in tumor progression [26]. We used qRT-PCR and western blot analysis to calculate EMT related genes expression, and we found that Vimentin and N-cadherin expression increased, but E-cadherin expression decreased (Figure 2F and 2G), which indicated DDR1 could activate EMT pathway.

Given the importance of glutamine metabolism in maintaining the malignancy of cancer cells [27], we measured DDR1’s effect on glutamine metabolism marker molecules. As shown in Figure 1G, upregulation of DDR1 increased the protein level of GLUD1 (glutamate dehydrogenase 1), GLS1 (glutaminase) and SLC1A (glutamate transporter). In addition, immunofluorescence results showed that the fluorescence intensity of GLUD1, GLS1 and SLC1A was higher in DDR1 overexpression cells than NC cells (Figure 2H and 2I). These data suggested DDR1 promoted HCC progression and glutamine metabolism, and activated EMT pathway.

RETRACTED

### Knockdown of DDR1 inhibits EMT and glutamine metabolism in SNU-182 cells

As shown in Figure 1D and 1E, DDR1 has the highest expression in SNU-182, and we transfected siRNA of DDR1 into SNU-182 cells to inhibit DDR1 expression (Figure 3A and 3B). Further functional experiments revealed that loss of DDR1 suppressed the proliferation, migration and invasion of SNU-182 cells (Figure 3C–3E). Meanwhile, knockdown of DDR1 decreased Vimentin and N-cadherin expression and increased E-cadherin expression (Figure 3F and 3G), which suggested si-DDR1 blocked EMT pathway. Deficiency of DDR1 also inhibited the expression of glutamine metabolism related molecules GLUD1, GLS1 and SLC1A (Figure 3H). Taken together, knockdown of DDR1 inhibited EMT and glutamine metabolism in HCC development.

**Figure 3:** **Loss of DDR1 inhibits EMT and glutamine metabolism in SNU-182 cells. The siRNA of DDR1 or NC was transfected into SNU-182 cells.** The expression of DDR1 was detected by qRT-PCR (**A**) and western blot (**B**) (n = 6, *p<0.05). (**C**) CKK-8 assay was used to examine cell growth at 0, 24, 48 and 72 h (n = 10, *p<0.05). (**D**) Wound healing assay was used to detect cell migration (n = 6, *p<0.05). (**E**) Transwell assay was performed to check cell invasion (n = 6, *p<0.05). qRT-PCR (**F**) and western blot (**G**) were used to test the expression of EMT related genes: Vimentin, N-cadherin and E-cadherin (n = 6, *p<0.05). (**H**) The protein expression of glutamine metabolism related genes: GLUD1, GLS1 and SLC1A was determined by western blot (n = 6, *p<0.05).

### DDR1 activates STAT3 pathway and interacts with STAT3

Due to STAT3 has dual functions of signal transduction and transcription regulation, we conjectured DDR1 participated HCC process by regulating STAT3 pathway. And we found the overexpression of DDR1 promoted the phosphorylation of STAT3 in tyrosine 705 and serine 727 in Hep3B cells (Figure 4A). Meanwhile, knockdown of DDR1 decreased the phosphorylation of STAT3 in SNU-182 cells (Figure 4B). CO-IP (co-immunoprecipitation) assay showed that DDR1 was coimmunoprecipitated with STAT3, and STAT3 was coimmunoprecipitated with DDR1 in HCC cells (Figure 4C), and there was a higher binding content in HCC tissues between DDR1 and STAT3 than that in adjacent tissues (Figure 4D). In addition, immunofluorescence analysis showed DDR1 bound with STAT3 in nucleus (Figure 4E). Because STAT3 is present in the cytoplasm and can be transferred to the nucleus to bind to DNA after activation, and we found a binding of DDR1 with STAT3 in nucleus. Thus, we wondered whether STAT3 could bind to the promoter region of DDR1. We used Jaspar (http://jaspar.genereg.net/) to predict the binding between STAT3 and DDR1 promoter (Table 1). Next, we used luciferase assay to test the binding between STAT3 and DDR1 promoter. And we found that the STAT3 increased the luciferase activity of WT DDR1 but not the mutant DDR1 (Figure 4F). Furthermore, overexpression of STAT3 increased the mRNA and protein expression of DDR1, while si-STAT3 showed the opposite effect (Figure 4G and 4H).

RETRACTED

**Figure 4:** **DDR1 interacts with STATA and promotes STAT3 phosphorylation.** (**A**) DDR1 plasmid or NC was transfected into Hep3B cells. Western blot was performed to test the expression of STAT3 and phosphorylated STAT3 (n = 6, *p<0.05). (**B**) The siRNA of DDR1 or NC was transfected into SNU-182 cells. The level of STAT3 and phosphorylated STAT3 was calculated by western blot (n = 6, *p<0.05). (**C**) CO-IP was used to determine the relationship between DDR1 and STAT3. DDR1 was pulled down by STAT3, and STAT3 was pulled down by DDR1 (n = 4). (**D**) CO-IP analysis for DDR1 and STAT3 in adjacent normal tissues and HCC tissues. (**E**) Immunofluorescence analysis used to detect the location of DDR1 and STAT3. Nucleus was blue stained by DAPI, red represents STAT3 and green represents DDR1. (**F**) Luciferase assay used to determine the binding between STAT3 and DDR1 promoter (n = 6, *p<0.05). STAT3 plasmid or siRNA of STAT3 or NC was transfected into Hep3B cells. The mRNA expression or protein level of DDR1 was tested by qRT-PCR (**G**) and western blot (**H**), respectively (n = 6, *p<0.05).

**Table 1:** Jaspar data of predicting the binding between STAT3 and DDR1 promoter.

**Matrix ID**	**Name**	**Score**	**Relative score**	**Sequence ID**	**Start**	**End**	**Strand**	**Predicted sequence**
MA0144.2	STAT3	6.98035	0.882118525	DDR1	1029	1039	-	GTGCTTGTAAT
MA0144.2	STAT3	6.63316	0.877912503	DDR1	1817	1827	-	CAGCAGGGAAA
MA0144.2	STAT3	4.01335	0.846174637	DDR1	1021	1031	+	GTGCTGGGATT
MA0144.2	STAT3	3.68262	0.842167999	DDR1	1650	1660	+	CTTCTGGACAT
MA0144.2	STAT3	3.62531	0.841473794	DDR1	1668	1678	+	GTGCCTGCAAA
MA0144.2	STAT3	3.62051	0.841415556	DDR1	1398	1408	+	CTGCCTGGAGT
MA0144.2	STAT3	3.10125	0.835124994	DDR1	1113	1123	-	AGGCTGGGAAT
MA0144.2	STAT3	3.04509	0.834444641	DDR1	1618	1628	+	TTGCTGGAACA
MA0144.2	STAT3	2.91247	0.832837947	DDR1	1822	1832	+	CTGCTGGGATC
MA0144.2	STAT3	2.2897	0.825293403	DDR1	935	945	-	CTATTAGAAAA
MA0144.2	STAT3	1.70079	0.818159017	DDR1	1617	1627	+	GTTGCTGGAAC
MA0144.2	STAT3	1.37564	0.81422002	DDR1	566	576	-	CTCCTTGGGAA
MA0144.2	STAT3	0.964762	0.809242395	DDR1	1617	1627	-	GTTCCAGCAAC
MA0144.2	STAT3	0.959256	0.80917569	DDR1	693	703	+	CTCCCGGGATG
MA0144.2	STAT3	0.935076	0.808882761	DDR1	1805	1815	-	CAGCTGCGAAG
MA0144.2	STAT3	0.911327	0.808595051	DDR1	1505	1515	+	CTGCCAGAACA
MA0144.2	STAT3	0.731142	0.806412196	DDR1	1755	1765	-	TGGCCAGAAAA
MA0144.2	STAT3	0.504659	0.803668454	DDR1	1090	1100	-	CAGCTTGGGAA
MA0144.2	STAT3	6.98035	0.882118525	DDR1	1029	1039	-	GTGCTTGTAAT
MA0144.2	STAT3	6.63316	0.877912503	DDR1	1817	1827	-	CAGCAGGGAAA
MA0144.2	STAT3	4.01335	0.846174637	DDR1	1021	1031	+	GTGCTGGGATT
MA0144.2	STAT3	3.68262	0.842167999	DDR1	1650	1660	+	CTTCTGGACAT
MA0144.2	STAT3	3.62531	0.841473794	DDR1	1668	1678	+	GTGCCTGCAAA
MA0144.2	STAT3	3.62051	0.841415556	DDR1	1398	1408	+	CTGCCTGGAGT
MA0144.2	STAT3	3.10125	0.835124994	DDR1	1113	1123	-	AGGCTGGGAAT
MA0144.2	STAT3	3.04509	0.834444641	DDR1	1618	1628	+	TTGCTGGAACA
MA0144.2	STAT3	2.91247	0.832837947	DDR1	1822	1832	+	CTGCTGGGATC
MA0144.2	STAT3	2.2897	0.825293403	DDR1	935	945	-	CTATTAGAAAA
MA0144.2	STAT3	1.70079	0.818159017	DDR1	1617	1627	+	GTTGCTGGAAC
MA0144.2	STAT3	1.37564	0.81422002	DDR1	566	576	-	CTCCTTGGGAA
MA0144.2	STAT3	0.964762	0.809242395	DDR1	1617	1627	-	GTTCCAGCAAC
MA0144.2	STAT3	0.959256	0.80917569	DDR1	693	703	+	CTCCCGGGATG
MA0144.2	STAT3	0.935076	0.808882761	DDR1	1805	1815	-	CAGCTGCGAAG
MA0144.2	STAT3	0.911327	0.808595051	DDR1	1505	1515	+	CTGCCAGAACA
MA0144.2	STAT3	0.731142	0.806412196	DDR1	1755	1765	-	TGGCCAGAAAA
MA0144.2	STAT3	0.504659	0.803668454	DDR1	1090	1100	-	CAGCTTGGGAA

RETRACTED

### DDR1 promotes the EMT of HCC cells by regulating STAT3

To investigate whether DDR1 is involved in HCC progression by regulating STAT3, we transfected siRNA of STAT3 into Hep3B cells, and qRT-PCR analysis showed a distinct decrease of STAT3 mRNA level in si-STAT3 transfected cells (Figure 5A). Then, we cotransfected DDR1 plasmid with or without si-STAT3 into Hep3B cells and found that silencing of STAT3 inhibited DDR1 expression (Figure 5B). Followed functional experiments showed that knockdown of STAT3 removed promoting effects of DDR1 on cell proliferation, migration and invasion (Figure 5C–5E). In addition, we explored the function of DDR1/STAT3 on EMT pathway and glutamine metabolism. The data suggested si-STAT3 decreased Vimentin and N-cadherin expression and increased E-cadherin expression, which was contrary to that in DDR1 transfected cells (Figure 5F and 5G). Likewise, loss of STAT3 inhibited the expression of glutamine metabolism related molecules GLUD1, GLS1 and SLC1A (Figure 5H). Together, DDR1 promoted EMT and glutamine metabolism in HCC cell by regulating STAT3.

**Figure 5:** **DDR1 promotes the EMT of HCC cells by regulating STAT3**. siRNA of STAT3 or NC was transfected into Hep3B cells, the transfection efficiency was tested by qRT-PCR (**A**) and western blot (**B**) (n = 6, *p<0.05). DDR1 was cotransfected into Hep3B cells with si-STAT3. (**C**) CCK8 assay was used to calculate cell proliferation (n = 10 *p<0.05). (**D**) Wound healing assay was used to detect cell migration (n = 6, *p<0.05). (**E**) Transwell assay was performed to check cell invasive ability (n = 6, *p<0.05). qRT-PCR (**F**) and western blot (**G**) were used to test the expression of EMT related genes: Vimentin, N-cadherin and E-cadherin (n = 6, *p<0.05). (**H**) The protein expression of glutamine metabolism related genes: GLUD1, GLS1 and SLC1A was determined by western blot (n = 6, *p<0.05).

RETRACTED

### Loss of DDR1 inhibits HCC progression by inactivating STAT3

To further explore the function of DDR1/STAT3 in HCC tumorigenesis, we set up xenograft nude mice model. Stable si-DDR1 or si-NC transfected SNU-182 cells were constructed (Figure 6A), and were subcutaneously injected in right lower limb of the nude mice. 1 week later, we injected lentivirus packaged STAT3 or NC into tumors. The tumors were isolated at 35 days after injection, si-DDR1 significantly decreased tumors weight, while overexpression STAT3 reversed si-DDR1 effect on tumors weight (Figure 6B). Furthermore, immunohistochemical results showed that si-DDR1 suppressed Ki67 expression, while injection of STAT3 promoted Ki67 level (Figure 6C). Knockdown of DDR1 inhibited DDR1 expression and STAT3 activation in tumors, while injection of STAT3 remitted the inhibitory role of DDR1 (Figure 6D). Intriguingly, tumors with si-DDR1 showed a decrease of Vimentin and N-cadherin and an increase of E-cadherin (Figure 6E and 6F), deficiency of DDR1 inhibited GLUD1, GLS1 and SLC1A expression (Figure 6G). Nevertheless, overexpression STAT3 promoted EMT and activated glutamine metabolism (Figure 6E–6G). Moreover, we performed tumor metastasis analysis, and found that loss of DDR1 inhibited tumor metastasis to lung, while overexpression of STAT3 removed the inhibitory effect (Figure 6H). These results indicated that knockdown of DDR1 inhibits HCC progression by suppressing activation of STAT3.

**Figure 6:** **Downregulation of DDR1 inhibits HCC progression by regulating STAT3 in nude mice.** Stable si-DDR1 or si-NC transfected SNU-182 cells were constructed (**A**) (n = 6, *p<0.05), and were subcutaneously injected into the right flanks of the nude mice. 1 week later, we injected lentivirus packaged STAT3 into tumors. (**B**) Tumor weight was determined in the isolated tumors from the nude mice (n = 4, *p<0.05). (**C**) Immunohistochemical staining of Ki67 used to determine cell proliferation (n = 4, *p<0.05 *vs* si-NC, ^#^*p*<0.05 *vs* si-DDR1). (**D**) Western blot analyzed the protein level of DDR1, p-STAT3 and STAT3 in tumors (n = 4, *p<0.05 *vs* si-NC, ^#^*p*<0.05 *vs* si-DDR1). qRT-PCR (**E**) and western blot (**F**) were used to test the expression of EMT related genes: Vimentin, N-cadherin and E-cadherin (n = 4, *p<0.05 *vs* si-NC, ^#^*p*<0.05 *vs* si-DDR1). (**G**) The protein expression of glutamine metabolism related genes: GLUD1, GLS1 and SLC1A was determined by western blot (n = 4, *p<0.05 *vs* si-NC, ^#^*p*<0.05 *vs* si-DDR1). (**H**) Stable si-DDR1 or si-NC transfected SNU-182 cells was intraperitoneally injected into mice, and lentivirus packaged STAT3 was injected into mice through tail vein 3 days later. Lungs were taken out and tumor numbers were calculated 4 weeks later.

RETRACTED

### STAT3 promotes HCC development by increasing DDR1

To explore the function of STAT3/DDR1 in HCC development, we constructed stable STAT3 or NC transfected Hep3B cells (Figure 7A). Cells were subcutaneously injected in right lower limb of the nude mice, and we injected lentivirus packaged si-DDR1 or si-NC into tumors at 7 days after injection. The tumors were isolated at 35 days after injection and were weighed. Overexpression of STAT3 expressively increased tumor weight comparing with NC group (Figure 7B). As well, STAT3 increased Ki67 expression, which indicated a promoting effect of STAT3 on HCC proliferation (Figure 7C). Overexpression of STAT3 inhibited DDR1 expression in isolated tumors, while silencing of DDR1 inhibited DDR1 protein level (Figure 7D). In addition, STAT3 promoted EMT of HCC which exhibited an increase of Vimentin and N-cadherin and a decrease of E-cadherin (Figure 7E and 7F). Forced expression of STAT3 accelerated GLUD1, GLS1 and SLC1A expression (Figure 7G). Interestingly, knockdown of DDR1 reversed the promoting effect of STAT3 on HCC progression. Comparing with STAT3 group, loss of DDR1 decreased tumor weight and Ki67 expression (Figure 7B and 7C), and knockdown of DDR1 inhibited EMT pathway and glutamine metabolism (Figure 7E–7G). Tumor metastasis analysis further indicated that STAT3 promoted tumor metastasis to lung, while silencing of DDR1 remitted the effect of STAT3 (Figure 7H). Taken together, STAT3 promoted HCC development by increasing DDR1.

**Figure 7:** **STAT3 promotes HCC development by increasing DDR1 in nude mice.** Stable STAT3 or NC transfected SNU-182 cells were constructed (**A**) (n = 4, *p<0.05), and were subcutaneously injected into the right flanks of the nude mice. 1 week later, we injected lentivirus packaged si-DDR1 into tumors. (**B**) Tumor weight was calculated (n = 4, *p<0.05). (**C**) Immunohistochemical staining for Ki67 (n = 4, *p<0.05 *vs* NC, ^#^*p*<0.05 *vs* STAT3). (**D**) Western blot analysis for DDR1 protein expression (n = 4, *p<0.05 *vs* NC, ^#^*p*<0.05 *vs* STAT3). qRT-PCR (**E**) and western blot (**F**) for EMT related genes expression: Vimentin, N-cadherin and E-cadherin (n = 4, *p<0.05 *vs* NC, ^#^*p*<0.05 *vs* STAT3). (**G**) Western blot analysis for protein expression of glutamine metabolism related genes: GLUD1, GLS1 and SLC1A (n = 4, *p<0.05 *vs* NC, ^#^*p*<0.05 *vs* STAT3). (**H**) Stable STAT3 or NC transfected SNU-182 cells was intraperitoneally injected into mice, and lentivirus packaged si-DDR1 was injected into mice through tail vein 3 days later. Lungs were taken out and tumor numbers were calculated 4 weeks later.

RETRACTED

## DISCUSSION

Hepatocellular carcinoma is one of the malignant tumors with the highest mortality, more than 600,000 deaths per year [28]. The lack of effective therapeutic targets is the main reason for the poor prognosis of HCC patients, thus exploring the potential pathogenesis of HCC has become a necessary method to prevent and treat HCC.

In the study of molecular mechanisms related to early recurrence of HCC, screening molecular targets closely related to the biological characteristics of HCC high invasion has become an important basis for targeted treatment of HCC [29, 30]. Our previous study used cDNA microarray and compared the difference between early recurrence and non-recurrence of early postoperative tumor tissue gene expression profiles of HCC, found DDR1 acted the key factor of early recurrence in HCC [9]. And in present study, we found a remarkable increase of DDR1 in HCC clinical tissues and cell lines. Furthermore, the expression of DDR1 was positively with the clinical grade of HCC, and low DDR1 expression patients had a higher 7-year survival rate.

Cancer is a metabolic disease, and energy metabolism restructuring is one of the important mechanisms to promote tumor progression [31]. Previous studies have suggested that mitochondrial oxidative and respiratory functions of tumor cells are defective, and tumor cells are powered by glycolysis [32]. However, recent studies have confirmed that mitochondrial oxidative respiratory function of tumor cells has not been lost [33, 34]. In some cases, tumor cells prefer to use glutamine metabolism to meet energy needs [35, 36]. Current research has confirmed that glutamine metabolism is a highly dependent metabolic pathway for HCC and is closely related to tumor progression [37]. Glutamine metabolism has become a new metabolic pathway for targeted metabolic therapy. And in present study, we found that upregulation of DDR1 promoted EMT and HCC cell progression. Further, the glutamine metabolism was also increased in DDR1 transfected cells, which indicated that DDR1 might promote HCC by upregulating EMT and glutamine metabolism. As expect, downregulation of DDR1 suppressed HCC progression by inhibiting EMT and glutamine metabolism.

RETRACTED

Current studies have proved that the binding of DDR1 with collagen promotes the activation of intracellular kinases, which then promotes the phosphorylation of downstream pathway proteins, and thus regulates multiple tumor signaling pathways [38]. And in our study, we found that overexpression of DDR1 increased the expression of STAT3, DDR1 also promoted the phosphorylation of STAT3. Further experiments showed that DDR1 colocalized with STAT3, which might be the potential mechanism of DDR1 activating STAT3. Considering the properties of STAT3 entering the nucleus and activating downstream molecules [39, 40], we predicted the binding of STAT3 with DDR1 promoter and there were 17 possible combination. regions. Then, the luciferase assay suggested that the STAT3 could bound with the promoter of DDR1. Overexpression of STAT3 increased the mRNA and protein expression of DDR1, while si-STAT3 showed the opposite effect. Furthermore, we found that DDR1 promoted the EMT and glutamine metabolism of HCC cells by upregulating STAT3. Meanwhile, in vivo tumor formation experiments proved that knockdown of DDR1 inhibits HCC progression by upregulating STAT3 and STAT3 promoted HCC development by increasing DDR1, which revealed the cross talk between DDR1 and STAT3 promoted the development of HCC by regulating EMT and glutamine metabolism.

## CONCLUSIONS

Our study suggested DDR1 and STAT3 formed a positive feedback pathway, synergistically promoted the progression of HCC, thus providing new evidence and new targets for the treatment of targeting glutamine metabolism in hepatocellular carcinoma.

## MATERIALS AND METHODS

### Clinical samples

Fresh cancer tissue samples and adjacent normal tissue samples were taken from 15 HCC patients undergoing surgical procedures at Guangdong Provincial People’s Hospital. We also collected HCC tissues from patients with tumor grade I (n = 8), grade II (n = 8) and grade III (n = 8). All of the patients or their guardians provided written consent, and this study was approved by the Ethics Committee of Guangdong Provincial People’s Hospital.

### Cell culture and treatment

The cell lines were purchased from the Science Cell Laboratory. Cells were cultured in RPMI 1640 (GIBCO, USA) supplemented with 10 % fetal bovine serum (Cromwell, USA) and 100 μL/mL penicillin and streptomycin (Sigma-Aldrich, USA) and placed at 37°C with 5% CO2. Cell transfection was performed as previous described [7]. Briefly, 2 μg plasmid or 500 nM si-RNA or its NC was transfected into cells with Lipofectamine^TM^ 2000 (Invitrogen, Carlsbad, CA, USA), respectively.

RETRACTED

### RNA isolation and qRT-PCR

RNA isolation, reverse transcription and quantitative expression were carried according to manufacturer’s instructions. All the kits were purchased from Vazyme, and gene expression was calculated using 2^-ΔΔCt^ method.

### Protein isolation and western blot

Total protein was collected from cells with RIPA lysis Mix. Western blotting assay was performed as previously described [23]. Briefly, 60 μg protein extractions were loaded via SDS-PAGE and transferred onto nitrocellulose membranes (absin, China), then incubated with primary antibodies for 2 hrs at temperature, then plated at 4 °C overnight, the membranes were incubated in 5% non-fat milk blocking buffer for horizontal mode 3 h. After incubation with secondary antibodies IRDye700/800 Mouse or Rabbit (Lincoln, Nebraska, USA), the membranes were scanned using an Odyssey, and data were analyzed with Odyssey software (LI-COR, USA). Primary antibodies list: DDR1 (SAB1300850, Sigma, USA), Vimentin (10366-1-AP, Proteintech, USA), N-cadherin (22018-1-AP, Proteintech, USA), E-cadherin (20874-1-AP, Proteintech, USA), GLUD1 (14299-1-AP, Proteintech, USA), GLS1 (12855-1-AP, Proteintech, USA), SLC1A5 (20350-1-AP, Proteintech, USA), STAT3 (10253-2-AP, Proteintech, USA), p-STAT3(705) (ab76315, Abcam, UK), p-STAT3(727) (ab32143, Abcam, UK), GAPDH (60004-1-Ig, Proteintech, USA).

### CCK8 assay

Cells were seeded in 96-well cell plates, and added CCK-8 (Cell Counting Kit-8) solution (Vazyme, China) at 0, 24, 48 and 72 h. 2 hours later, measure the OD value at 450 nm.

### Wound healing assay

5×10^5^ cells were planted in a 6-well plate, and when the cells grew to fuse, two vertical parallel lines were drawn with 10 μL suction head against the ruler. The floating cells were washed with PBS and cultured in serum-free medium for 24 hours. Images were taken at 0 and 24 hours of cell culture, respectively.

### Transwell assay

Cells in logarithmic growth phase were adjusted to 2 × 10^5^ cells/well of medium (without serum) and plated into the upper chamber insert pre-coated with 1μg/μl Matrigel. Lower chamber was added with 500 μL of medium (with 10% FBS), and then incubate the chamber at 37°C for 48 h. Then the invading cells were visualized by the crystal violet and inverted microscope.

### In vivo tumor growth and metastasis assay

Nude mice were purchased from Guangdong provincial experimental animal center for medicine. Tumor growth assay: Stable si-DDR1 or STAT3 transfected SNU-182 (5 x 10^6^) were subcutaneously injected in right lower limb of the nude mice, and lentivirus packaged STAT3 or si-DDR1 was injected into tumors 1 week later. Tumor size was measured every five days. After 30 days of injection, the tumor was removed for follow-up study. Tumor metastasis assay: Stable si-DDR1 or STAT3 transfected SNU-182 cells was intraperitoneally injected into mice, and lentivirus packaged STAT3 or si-DDR1 was injected into mice through tail vein 3 days later. Lungs were taken out and tumor numbers were calculated 4 weeks later.

RETRACTED

### Immunofluorescence staining

Cells were plated in a 24-well cell culture plate. After transfection, cells were washed by PBS and fixed with 4% paraformaldehyde. Cells were permeabilized with 0.2% Triton-X-100 solution in PBS. Next, we blocked cell using goat serum. Then, the cells were incubated with GLUD1, GLS, SLC1A5 antibody at 4 °C overnight followed with FITC-conjugated goat anti-mouse antibodies incubation for 1h. After three washes with PBS, we incubated cells by DAPI (4',6-Diamidino-2-phenylindole, dihydrochloride).

Frozen sections of tumor tissue were fixated in 4% paraformaldehyde and washed using PBS. We penetrated sections using 0.5% Triton X-100. After 3 times wash, we blocked sections with 50% goat serum. Then, sections were incubated with Ki67 antibody overnight. We incubated the sections using secondary antibody followed by DAPI staining. Immunofluorescence was analyzed under an IX73 fluorescence microscope (Olympus, Valley, PA).

### Co-immunoprecipitation (CO-IP)

CO-IP assay was performed using Thermo Pierce Co-Immunoprecipitation Kit (Thermo, USA) according to the instruction. Briefly, cells were plated in a 6-well cell culture plate. After transfection, cells were washed by PBS and lysed by RIPA Buffer. And the agarose beads were added into total cell protein placed at 4°C shaking for 10 min. Then, the agarose beads were incubated with DDR1 or STAT3 antibody at 4°C overnight followed by western blot analysis.

### Luciferase assay

According to the Jaspar data, we mutated the bases from 1021-1031, 1650-1660, 1668-1678 and 1398-1408 in DDR1 promoter sequence (shown in supplementary materials). And the mutant DDR1 were synthesized by Invitrogen (Carlsbad, CA, USA). psiCHECK-2 luciferase reporter plasmid was inserted with the wild type DDR1 5’UTR or mutant DDR1 5’UTR sequences, then were transfected with reporter vectors into HEK293 cells. The cells were collected after 48 h post-transfection and lysed to detected the luciferase activity (Promega). The promoter sequence of DDR1 was shown in supplementary materials. And mutant DDR1 was mutated the binding bases of DDR1 to STAT3.

### Statistical analysis

Results are expressed as mean values ± standard deviation. Statistical analyses were assessed with Student’s test and one-way ANOVA using GraphPad Prism 7.0 and SPSS19.0. P values of less than 0.05 were considered significant.

RETRACTED

## Supplementary Material

Supplementary Materials
